The article "On-Site Solid Waste Handling Practice and Associated Factors among Condominium Residents in Gondar City, Northwest Ethiopia, 2021: A Community-Based Cross-Sectional Study" was published in 2023. Journal: J Environ Public Health.

# On-Site Solid Waste Handling Practice and Associated Factors among Condominium Residents in Gondar City, Northwest Ethiopia, 2021: A Community-Based Cross-Sectional Study

**DOI:** 10.1155/2023/5267790

**Published:** 2023-01-28

**Authors:** Alemtshay Shiferaw, Nuhamin Tesfa Tsega, Amare Alemu, Mastewal Endalew, Bikes Destaw Bitew

**Affiliations:** ^1^Department of Environmental Health, College of Medicine and Health Sciences, University of Gondar Comprehensive Specialized Hospital, Gondar, Ethiopia; ^2^Department of Women's and Family Health, School of Midwifery, College of Medicine and Health Sciences, University of Gondar, Gondar 6200, Ethiopia; ^3^Ethiopian Public Health Institute, Addis Ababa 1000, Ethiopia; ^4^Department of Environmental and Occupational Health and Safety, Institute of Public Health, College of Medicine and Health Sciences, University of Gondar, Gondar 6200, Ethiopia

## Abstract

**Background:**

Solid waste is one type of waste that is released from human day-to-day activities and it is considered useless or unwanted for further use. Population growth, rapid urbanization, a booming economy, and an increase in the standards of living of the community have substantially enhanced the rate of solid waste generation in developing countries. Solid wastes can be used as a resource for industrial production or energy generation. However, it causes environmental and human health problems due to poor management. There is scanty information about on-site solid waste management practice in the study area. Therefore, assessing on-site solid management practices and their associated factors, especially for condominium residents is very important.

**Objective:**

To assess on-site solid waste handling practice and its associated factors among condominium residents in Gondar city, northwest Ethiopia, 2021.

**Methods:**

A community-based cross-sectional study was conducted from March 1 to June 15/2021 among condominium residents in Gondar city. The study included a total of 450 condominium households, with a 99.3% response rate. A binary logistic regression model was used to assess the association between dependent and independent variables. Those variables which have a *p* value <0.25 in the bivariate analysis were entered into a multivariable logistic regression model. A *p* value of less than 0.05 with 95% CI was considered a statistically significant factor.

**Result:**

In this study, 79.8% with 95% CI (76.4%, 83.3%) of condominium residents had poor on-site solid waste handling practices. The finding also showed that 42.2% and 50.2% of study participants have favorable attitudes and good knowledge towards on-site solid waste handling practices, respectively. In multivariable logistic regression analysis, male household heads (AOR = 1.90; 95% CI, 1.11–3.28), large family size (AOR = 1.87; 95% CI, 1.03–3.40), negative attitude towards on-site solid waste handling practices (AOR = 1.79; 95% CI, 1.07–3.00), not receiving training (AOR = 3.40; 95% CI, 1.77–6.55), and not having legal enforcement (AOR = 2.85; 95% CI, 1.39–5.84) were significantly associated with on-site solid waste handling practices.

The article "On-Site Solid Waste Handling Practice and Associated Factors among Condominium Residents in Gondar City, Northwest Ethiopia, 2021: A Community-Based Cross-Sectional Study" was published in 2023. Journal: J Environ Public Health.

**Conclusion:**

The on-site solid waste handling practice of condominium households was very poor. The provision of training and enforcement of rules regarding solid waste handling is necessary.

## 1. Background

Solid waste is defined as any garbage or refuse and other discarded material that has no further use or value for the person or organization that owns it and which will be discarded [1, 2]. On-site solid waste handling practice refers to the separation, storing, collection, reusing or recycling, processing, and preparing for final disposal of solid wastes until the waste is placed in the solid collection bin used for storage before collection [3]. The main constituents of residential solid waste in urban areas are organic waste, paper, glass, metals, and plastics, and ash and dust are a significant portion of the waste [4].

In 2016, the world's cities generated 2.01 billion tons of solid waste, accounting for 0.74 kilograms per person per day [5]. By 2050, worldwide municipal solid waste generation is expected to have increased to 3.4 billion metric tons [5]. In low-income countries, over 90% of waste is often disposed of in unregulated dumps or openly burned [5]. In developing countries, dumping solid waste in the yard and throwing it in the ditch and the river are a common activity [6]. Furthermore, in least-developed countries such as Ethiopia, an estimated 30 to 50% of solid waste produced in the urban area is left uncollected [7]. In Ethiopia, the average municipal solid waste generation rate ranges from 0.25 to 0.49 kg/capita/day [8]; moreover, it is not properly managed. This is due to the increase in the national population, the rising demand for food, urbanization, economic growth, and the improved lifestyle of people, which results in the increased generation of solid wastes in urban as well as rural areas of the country [9]. An increase in waste generation rate is a challenge to handle solid waste properly nowadays. As a result, poor solid waste handling causes human and environmental health problems [10]. In a study conducted in Asella town, Ethiopia, about 72.8% of respondents did not separate solid waste at source [6]. Most of the solid waste is not separated by households because of a lack of awareness and in some cases negligence [11]. Solid waste management in Ethiopia has focused only on dumping, and managing it at the point of generation is not known [12]. Out of the total waste generated in different cities of Ethiopia, 67.4% is organic biodegradable waste [12]. Because of the lifestyle change, the current composition of solid waste in Ethiopia has increased its proportion of plastics and packaging materials [13]. Poor solid waste management has the potential to attract disease-carrying vectors. Insect and rodent vectors can also breed in solid waste. Open burning of solid wastes results in the emission of noxious gases and causes water source pollution due to the open dumping of toxic wastes. In addition, in urban areas, waste dump is the cause of aesthetic problems, challenging traffic and reducing the beauty of the city [14].

The article "On-Site Solid Waste Handling Practice and Associated Factors among Condominium Residents in Gondar City, Northwest Ethiopia, 2021: A Community-Based Cross-Sectional Study" was published in 2023. Journal: J Environ Public Health.

Due to differences in lifestyle, consumption pattern, and income level, urban residents are generating a high amount of waste than rural areas. The rapid population growth in urban areas has created difficulties for local authorities to adequately provide waste management services in developing countries [15]. Nowadays, the government of Ethiopia is appreciating the condominium type of infrastructure to solve residential housing problems in urban settings, because condominiums can house a large number of people in a limited amount of space. However, it may be challenging to handle waste safely because of overcrowded settlements [16].

Implementing the management principles such as waste reduction, reuse, and recycling is not prioritized by the municipalities for sustainable solid waste management [7]. This is mainly due to inadequate institutional capacity, finances, lack of knowledge, weak political commitment and prioritization, and a lack of effective planning and implementation [12].

The Ethiopian government has previously adopted solid waste management policies and legal frameworks to reduce the environmental and human health impacts caused by poor solid waste handling practices [8]. However, it is not implemented due to a lack of enforcement. Even the problem makes it difficult to achieve Sustainable Development Goal 6: “improving water quality by reducing pollution, eliminating dumping, and minimizing release of hazardous chemicals and materials, halving the proportion of untreated wastewater, and substantially increasing recycling and safe reuse globally.” Proper on-site solid waste handling practices require the commitment of the city's sanitation and beautification (SB) office and the active involvement of the community members. Although Gondar city has a formal sanitation and beautification (SB) office, it is ineffective in solid waste management due to a variety of factors [7]. As a result, the sanitary conditions of the city have become a threat from time to time to both human health and the environment, and residents are suffering from living in such a holistic environment. Gondar city was in a difficult geographical location. Currently, the city's population is increasing on a regular basis. To address this issue, residents are given condominium-style housing, because it can house a large number of people in a small area. In comparison to other residential areas, on-site solid waste management practice among condominium residents is difficult. To begin with, because most condominium residents pay rent and many people share a building, people may lack responsibility for the building's hygiene. Second, the majority of condominium residents are educated, and residents are relatively wealthy, as the amount and type of solid waste differ from the general population. Third, condominium residents who live in an overcrowded environment lack streets between buildings and have waste storage site problems.

The article "On-Site Solid Waste Handling Practice and Associated Factors among Condominium Residents in Gondar City, Northwest Ethiopia, 2021: A Community-Based Cross-Sectional Study" was published in 2023. Journal: J Environ Public Health.

Therefore, this study was determined on-site solid waste handling practices and associated factors among condominium residents in Gondar city. The findings of the study could help local policymakers to develop problem-solving policies. It could help for the city's sanitation and beautification as a source of information to implement and prioritize their activities based on identified factors.

## 2. Methods and Materials

### 2.1. Study Design and Period

A community-based cross-sectional study design was used to study on-site solid waste handling practices among condominium residents from March 1 to June 15/2021.

### 2.2. Study Area

The study was conducted on Gondar city condominium residents. Gondar city is located 727 km from Addis Ababa, 175 km from Bahir Dar, and 120 km from the Simien Mountains. In the city, the famous Gondar castles of Ethiopia are found and now being part of the United Nations Educational, Scientific and Cultural Organization (UNESCO) World Heritage Site [17]. Other structures in and around the city that are part of the UNESCO World Heritage Site are Fasil Ghebbi, Fasilides' Bath, Qusquam Enclosure, and the Epiphany. These historical places attracted many visitors across the world. With a population of more than 200,000 inhabitants, Gondar is growing rapidly due to fast urbanization, like all other cities in Ethiopia [17]. The rapid expansion in population has resulted in increased volumes of solid trash and, as a result, increased infrastructure demand. The majority of solid waste created in the city goes uncollected and is simply thrown in open spaces, roadsides, river courses, and gullies [7]. The nature of the topography of Gondar has a great influence on the development of the city, since the major portion of the topography comprises scattered hills, valleys, and eroded lands [7]. The city has five condominium residence villages with 2,419 households.

The article "On-Site Solid Waste Handling Practice and Associated Factors among Condominium Residents in Gondar City, Northwest Ethiopia, 2021: A Community-Based Cross-Sectional Study" was published in 2023. Journal: J Environ Public Health.

### 2.3. Source and Study Population

All five condominium households in Gondar city were the source of population, whereas all selected households in the condominium villages were the study population.

### 2.4. Sample Size Determination and Sampling Procedures

The sample size was determined based on the two objectives. The sample size for the first objective was calculated by using a single population proportion formula, *n* = (*Z*_*α*/2_)^2^*P*(1 − *P*)/*d*^2^), considering the following assumption: proportion of proper on-site solid waste handling practices was 23.9% in Debre Markos town among condominium residents [18], a 95% confidence level (*Z* = 1.96), and 5% margin of error. Therefore, *n* = (1.96)^2^ 0.239(1–0.239)/0.05^2^)) = 279. So, the minimum sample size (*n*) after adding a 15% nonresponse rate was 321 households.

The sample size for the second objective was calculated using Epi Info version 7 with an assumption of 95% confidence level, 80% power, and 5% margin of error, taking into account monthly income, the number of solid waste storage containers, campaign participation level, perceptions on hygiene policy enforcement and responsibility, and access of streets between buildings as a factor from a previous study conducted in Debre Markos town [18]. The final sample size was 453 after adding a 15% expected nonresponse rate, which was obtained from the access of streets between building factors because it provides the largest sample size when compared to other factors and the first objective.

The Amhara building construction agency registered condominium households, and each condominium household was assigned a number beginning with one. First, the study households were allocated proportionally based on the number of sites in the five condominiums, namely, Azezo site (233 from 1246 HHs), Aba Samuel site (101 from 540 HHs), College site (93 from 496 HHs), Gibrna site (19 from 98 HHs), and Awura Godana site (7 from 39 HHs). The 453 households were then chosen using simple random sampling methods by providing identification codes ranging from 1 to 2429 HHs.

### 2.5. Operational Definitions

#### 2.5.1. On-Site Solid Waste Handling Practice

In this study, participants who scored less than or equal to the mean value of 12 on-site solid waste handling practice items were considered as having poor practices and those participants who scored greater than the mean value were considered as having good practices [18].

The article "On-Site Solid Waste Handling Practice and Associated Factors among Condominium Residents in Gondar City, Northwest Ethiopia, 2021: A Community-Based Cross-Sectional Study" was published in 2023. Journal: J Environ Public Health.

#### 2.5.2. Knowledge

In this study, participants who scored less than or equal to the mean value of eight on-site waste handling-related knowledge questions were considered as having “poor knowledge” and those participants who scored greater than the mean value were considered as having “good knowledge” [19, 20].

#### 2.5.3. Attitude

In this study, participants who scored less than or equal to the mean value of seven on-site solid waste handling-related attitude questions were considered as having “unfavorable attitude” and those participants who scored greater than the mean value were considered as having “favorable attitude” [19–21].

#### 2.5.4. Condominium

It means an apartment (building) constructed by the government or a private company with shared walls and corridors [18].

### 2.6. Data Collection Tool and Processes

The data were collected by face-to-face interviews with adult members of households (especially women whose age is above 18 years). Four BSc environmental health professionals and two supervisors were recruited for data collection and close supervision, respectively. The questionnaires were adapted and customized from different literatures [18–21]. The questionnaires had four sections including socio-demographic variables, knowledge, and attitude, infrastructural factors, and on-site solid waste handling practice items. The first section contains socio-demographic characteristics such as age, sex, marital status, educational status, occupation, religion, household income, family size, occupation, homeownership, and services of houses.

The second section contained knowledge of on-site solid waste handling practice-related questions such as knowledge on how to handle solid wastes, knowledge on reduction of solid waste at source, knowledge about solid waste reuse, knowledge of solid waste recycling, knowledge of human and environmental health problems related to poor solid waste handling, knowledge on potential contamination of water by solid wastes, and knowledge about personal protective equipment used to handle solid waste. After computing the sum of all items, knowledge was categorized as “poor” if the participants had less than equal to the mean value and “good,” otherwise. It was coded as “0” for poor knowledge and “1” for good knowledge of condominium residents.

The third section includes questions related to the attitude of participants towards on-site solid waste handling practices such as believing that each person should manage his/her waste, believing that inappropriate solid waste disposal can cause air pollution, believing that inappropriate solid waste management can cause health problem, believing that it is my responsibility to separate solid waste, believing that waste recycling is very important and being positive to reduce the amount of solid waste that produced, and believing that proper handling of solid waste can save money. In the same way to the knowledge of participants, the items of attitude were computed and classified based on the median value and it was coded as “0” for poor attitude and “1” for good attitude of condominium residents. The fourth section's institutional factors include access to streets to solid waste collectors, training regarding on-site solid waste handling practices, type of solid waste storage container provided, the existence of legal control over a society, and budget allocation for solid waste (SW) disposal.

The article "On-Site Solid Waste Handling Practice and Associated Factors among Condominium Residents in Gondar City, Northwest Ethiopia, 2021: A Community-Based Cross-Sectional Study" was published in 2023. Journal: J Environ Public Health.

The last section contains the on-site solid waste handling practices of participants which include separating solid waste at home, reusing solid waste at home, recycling solid waste at home, storing solid wastes, frequency of solid waste collection per week, dumping solid waste on the road, dumping solid waste on the ditch, dumping solid waste in the yard, burning SW in the compound, keeping SW far from food, keeping SW far from water, and keeping SW far away from children's playgrounds. After computing, the sum of all practice items and on-site solid waste handling practices were categorized as “poor” if the participants had less than equal to the mean value and “good,” otherwise. It was coded as “0” for good practices and “1” for poor practices of participants. To enhance the reliability of this data, self-report practices of households were supported through observation during the interview.

### 2.7. Data Quality Control

The questionnaire's quality was ensured by careful design, translation, and retranslation. Pretests were carried out on 5% of questionnaires in Debre Tabor town condominium residents, which have similar characters in the study area. One day of training was given for data collectors and supervisors regarding the content of questionnaires, way of communication, the value of confidentiality, and participant rights. The supervisors and principal investigator had close follow-up on a day-to-day basis to ensure the completeness and consistency of the collected data. Following that, proper categorization and coding of the data were performed.

### 2.8. Data Management and Analysis

Completed data were entered into Epi Info version 7 and then the data were exported into SPSS version 20 software for further analysis. Descriptive statistics mean with standard deviation (SD) or median with interquartile range (IQR) values were used to present continuous data, as well as the percentage and frequency tables for categorical data. The model fitness was checked by using the Hosmer and Lemeshow test which revealed a *p* value of 0.21. Associations between independent variables were checked by multicollinearity test and all variables had variance inflation factor (VIF) value less than 2. Bivariate logistic regression analysis was performed and selected variables (with a *p* value below 0.25) were candidates for multivariable logistic regression. After controlling for confounders, multivariable analysis results were expressed as adjusted odds ratios (OR). Results with a *p* value of less than 0.05 and 95% CI were declared statistically significant associated factors.

The article "On-Site Solid Waste Handling Practice and Associated Factors among Condominium Residents in Gondar City, Northwest Ethiopia, 2021: A Community-Based Cross-Sectional Study" was published in 2023. Journal: J Environ Public Health.

## 3. Results

### 3.1. Socio-Demographic Characteristics of Study Participants

A total of 450 study participants were involved in this study, with a response rate of 99.3%. More than half (57.1%) of the study participants were females. The median age of respondents was 34 years (IQR = 11 years). About 295 (65.6%) respondents were married and 299 (66.4%) were orthodox religion followers. Regarding education status, about 47 (10.4%) of respondents had no formal education, whereas more than half (60.4%) of study participants had a diploma and above. More than three-fourths of households (69.8%) had less than five family members. Slightly below half of the study participants (46.7%) were employed in government sectors. The median monthly income of households was 7000 Ethiopian Birr (ETB) with IQR = 4000 ETB. Nearly two-thirds of residents (63.8%) live in rented houses (Table 1).

### 3.2. Knowledge of Condominium Residents towards On-Site Solid Waste Handling

In this study, 226 (50.2%) household heads had good knowledge regarding on-site solid waste handling. The majority of participants (77.6%) knew solid waste reduction at home, 85.3% knew solid waste reuse, and 80.7% knew that solid wastes can be recycled to create new products. The majority of respondents (90%) and 373 (82.9%) knew human health and environmental health problems related to poor on-site solid waste handling practices, respectively. About 412 (91.6%) of respondents knew the personal protective equipment used to handle solid wastes (Table 2).

### 3.3. The Attitude of Condominium Residents towards On-Site Solid Waste Handling Practices

In this study, only 191 (42.4%) study participants (heads of households) had a favorable attitude towards on-site solid waste handling practice. A small number of participants (10.4%) disagreed that poor solid handling practices can cause human health problems. Less than a quarter of respondents (13.8%) agreed that each person should manage his/her waste but the majority of respondents (94.0%) agreed that their responsibility separates the waste generated from the house. Moreover, three-fourths (79.3%) of participants said solid waste recycling was important. In addition, 84.4% of respondents believed that proper handling of solid waste can save money (Table 3).

The article "On-Site Solid Waste Handling Practice and Associated Factors among Condominium Residents in Gondar City, Northwest Ethiopia, 2021: A Community-Based Cross-Sectional Study" was published in 2023. Journal: J Environ Public Health.

### 3.4. Infrastructural and Institutional Related Factors

Nearly one-tenth (10.9%) of households had received training regarding on-site solid waste handling practices. About 67.3% of household heads reported that there was legal control over the community to keep good waste handling practices. Almost all (99.3%) condominium residents had access to the street to collect solid waste. The infrastructural and institution-related factors of condominium residents are summarized in Table 4.

### 3.5. On-Site Solid Waste Handling Practices

In this study, 79.8% with 95% CI (76.4, 83.3) of households followed poor on-site solid waste handling practices. The majority (83.8%) of households were separated from solid waste in their home. Only a few numbers of households (7.6%) reused solid wastes and 9.3% recycled solid wastes. About 12.9% of households damped solid waste on the road, on the ditch (5.8%), and in the yard (6.2%) (Table 5). In terms of solid waste generation type, food waste accounted for 87.1%, followed by plastic waste at 10.2%. Other wastes including old papers and anal cleaning materials from the toilet contained few numbers (Figure 1).

### 3.6. Factors Associated with Household On-Site Solid Waste Handling Practices

In bivariate analysis, variables such as age, sex, monthly household income, educational status, occupational status, family size, knowledge, attitude, training, and legal enforcement were significantly associated with poor on-site solid waste handling practices at a *p* value less than 0.25.

In multivariable analysis after adjusting ten variables, sex, family size, attitude, training, and legal enforcement have remained significant at a *p* value less than 0.05. The odds of poor solid waste handling practice were nearly 2 times more likely among males than their counterparts (AOR: 1.90; 95% CI: 1.1, 3.28). Condominium residents having large family members were 1.87 times more likely to have poor on-site solid waste handling practices than households with small family members (AOR: 1.87; 95% CI: (1.03, 3.40)). Respondents with unfavorable attitudes were 1.8 times more likely to follow poor on-site solid waste handling practice than their counterparts (AOR: 1.79; 95% CI: 1.07, 3.00). The odds of poor solid waste handling practices were 3.4 times higher among households who did not receive training towards on-site solid waste handling practices compared to those who received training (AOR: 3.40; 95% CI: 1.77, 6.55). The likelihood of poor on-site solid waste handling practices was reported about 2.9 times more likely among households who did not receive legal enforcement than their counterparts (AOR: 2.85; 95% CI: 1.39, 5.84). Factors associated with household on-site solid waste handling practice of condominium residents in Gondar city are summarized in Table 6.

The article "On-Site Solid Waste Handling Practice and Associated Factors among Condominium Residents in Gondar City, Northwest Ethiopia, 2021: A Community-Based Cross-Sectional Study" was published in 2023. Journal: J Environ Public Health.

## 4. Discussion

Solid waste, which is a byproduct of human activity, must be properly managed. The purpose of this study was to identify the main factors that influenced on-site solid waste handling practices, particularly among condominium residents. Since Gondar has many problems associated with a poorly managed solid waste system. In this study, 79.8% with 95% CI (76.4, 83.3) of condominium residents had poor on-site solid waste handling practices. This finding is in line with a study conducted in Asella town, central Ethiopia, 82.8% [6]. The current finding is also slightly higher than a study finding in Debre Markos town at 76.1% [18], in Nigeria 66.3% [22]. However, it is much higher than in Ghana 39.0% [23] and 59% in Thailand [24]. In contrast, the current finding is extremely lower than the studies conducted in Debre Birhan town, 91.5% [3]. The possible reason for this discrepancy might be the difference in the socio-economic status of the residents such as household income and educational level. Moreover, there might be also a difference in policy enforcement for the proper handling of solid wastes. Poor on-site solid waste management practices can have serious environmental consequences such as infectious diseases, land and water pollution, drain obstruction, and a loss of city beauty. The study's findings indicated that achieving Sustainable Development Goal 6, target 6.1, which is to provide the community with access to high-quality, safe drinking water services, is difficult. Poor on-site solid waste management systems, on the other hand, will be improved if condominium residents have access to modern sanitation systems as a result of meeting sustainable development goals.

The finding also revealed that 50.2% of respondents have good knowledge of solid waste handling practices which is lower than other studies conducted in Ethiopia, 81.8% [25], and Somalia, 58.0% [26], whereas 42.2% of study participants have a favorable attitude towards on-site solid waste handling practices and it is lower than other studies, 62.0% in Somalia [26] and 77.5% in another part of Ethiopia [25]. The level of good practices in this study was 20.2% and lower than in other studies conducted in Somalia, 35.0% [26]. The possible difference might be the variation in the educational level of the participants. Knowledge of solid waste disposal practices may be one of the most important determinants shaping a community's attitude and practice.

The article "On-Site Solid Waste Handling Practice and Associated Factors among Condominium Residents in Gondar City, Northwest Ethiopia, 2021: A Community-Based Cross-Sectional Study" was published in 2023. Journal: J Environ Public Health.

In our study, 83.8% of household heads were separated from solid wastes. In contrast, the majority (90.7%) of condominium residents in Debre Markos town did not separate solid wastes [18]. The separation of waste in this study was greater than in a study conducted in Kampala 49.7% [27]. In the current study, few households reused solid waste (7.4%) and recycled solid waste at home (9.3%). This finding is lower than the study conducted from Assela, Ethiopia, 10.5% [6], and slightly higher in the Debre Markos study (6.40%) [18]. Moreover, in this study, the majority (92.8%) of households did not separate solid waste at home, which is greater than the studies conducted in Debre Markos (90.7%) [18]. The possible difference might be variations in accessibility market access for separated solid wastes and in the attitude of participants to improve further solid waste management steps and the legal enforcement difference across the settings.

In this study, male residents experienced poor solid waste handling nearly 2 times more than their counterparts. This implied that solid waste handling at the household level was mainly the responsibility of the women compared with men [3, 27–29]. However, a contradicting finding in another study [30] is that solid waste management practices did not vary between male and female respondents. In the case of Ethiopia, females are responsible for every activity of the household; as a result, they may know the characteristics of each solid waste. Moreover, females give more emphasis to the cleanliness of their homes and the environment. Our study highlights the importance of gender-fair campaigns and other related programs relevant to addressing human and environmental health problems.

Household family size was significantly associated with on-site solid waste handling practices, whereas those household heads with five to eight family members had poor on-site solid waste handling practices. The number of household members increasing the waste generated at the household level would be higher and may initiate improper handling of wastes including disposing of wastes in a place where they can easily reach them without regard for the suitability of the disposal site. This study suggests that having a large number of household members may provide an opportunity to divide and complete tasks in solid waste management practice.

The article "On-Site Solid Waste Handling Practice and Associated Factors among Condominium Residents in Gondar City, Northwest Ethiopia, 2021: A Community-Based Cross-Sectional Study" was published in 2023. Journal: J Environ Public Health.

In this study, low enforcement of rules and regulations of the condominium site was significantly associated with poor solid waste handling practices. The finding is in line with studies conducted in Debre Markos town [18]; respondents had poor solid waste handling practices without legal enforcement. Even though Gondar city has rules and regulations that emphasized solid waste handling practices, low enforcement existed, as well as the majority of the city residents did not know the city rules and regulations regarding solid waste management [7]. Poor enforcement of rules and regulations may lead to harmful and illegal waste disposal methods because less attention is given to the area.

In addition, an unfavorable attitude was significantly associated with poor solid waste handling practices. This finding was supported by studies conducted in Thailand [24] and the Philippines [30], where a person with a good attitude also had good practices. People's attitudes influenced their choice of reusable things from the market over simple disposable items [30]. Our finding also confirmed that only a few respondents reused solid wastes due to poor attitudes towards solid waste handling practices. Households' attitude or view about solid waste collectors and their services is important for their service delivery performance [29]. Every household is expected to accept the idea that everyone is responsible for collecting and disposing of their solid waste.

In our study, training in solid waste handling was significantly associated with solid waste handling practices. Training, such as education and other sources, is a source of knowledge. As a result, people with higher knowledge scores were more likely to exhibit good practice in solid waste management [30]. Our study implies that information through training is necessary to improve on-site solid waste handling practices. A report from a Philippines study showed that the reuse of solid wastes including plastic/glass bottles, cans, paper, and rainwater was also associated with good knowledge of a person [30]. Therefore, training households about how to handle solid waste at the source of generation is very important.

### 4.1. Strength of the Study

We collected the most common types of condominium solid waste. Using a simple random method could increase the representativeness of the finding.

### 4.2. Limitation of the Study

We used a cross-sectional study design and the appropriateness of each solid waste handling practice in each day is not observed.

## 5. Conclusion

In this study, poor on-site solid waste handling practice of households was very high. Only some residents were reusing and recycling solid wastes. Respondents' overall knowledge and attitude toward on-site solid handling practices were low when compared to other areas. In this study, the sex of the household heads, household family size, attitude towards solid waste handling practices, training, and legal enforcement were the main determinates of poor solid handling practices. The Gondar city sanitation and beautification (SB) office should develop an awareness creation program emphasizing the importance of good on-site solid waste handling practices for the future solid waste management system and public health. Furthermore, the Gondar city health office should provide on-site solid waste handling method training for Health Extension Workers. In the back, Health Extension Workers should once again teach residents how to separate, reuse, and recycle solid waste at the household level. Lastly, the implementation of rule and regulation practicality is needed from Gondar city municipal.

The article "On-Site Solid Waste Handling Practice and Associated Factors among Condominium Residents in Gondar City, Northwest Ethiopia, 2021: A Community-Based Cross-Sectional Study" was published in 2023. Journal: J Environ Public Health.

## Figures and Tables

**Figure 1:** The common types of solid wastes generated from condominium households.

**Table 1:** Socio-demographic characteristics of condominium residents in Gondar city, northwest Ethiopia, 2021 (*n* = 450).

Characteristics	Categories	Frequencies	Percentages (%)
Age	<29	121	26.9
	29–34	108	24.0
	35–40	128	28.4
	>41	93	20.7

Sex	Male	212	47.1
	Female	238	52.9

Marital status	Single	137	30.4
	Married	295	65.6
	Divorced/windowed	18	4.0

Educational status	No formal education	52	11.6
	Formal education	398	88.4

Religion	Orthodox	299	66.4
	Muslim	125	27.8
	Protestant	26	5.8

Occupation	Gov't employee	210	46.7
	Private work	99	22.0
	Housewife	141	31.3

Household income (ETB)	<5000	150	33.3
	5000–7000	137	30.4
	7001–9000	95	21.1
	>9001	168	15.1

Family size	1–4 members	314	69.8
	5–8 members	136	30.2

Home ownership	Rented	287	63.8
	Private	163	36.2

Services of houses	For residence	310	68.9
	For commercial	140	31.1

**Table 2:** Knowledge of condominium residents towards on-site solid waste handling practices in Gondar city, northwest Ethiopia, 2021.

Question items	Categories	Frequencies	Percentages (%)
Know how to handle solid waste at home	Yes	293	65.1
	No	157	34.9

Know solid waste reduction at the source	Yes	349	77.6
	No	101	22.4

Know reuse of solid waste	Yes	384	85.3
	No	66	14.7

Know that solid waste can be used as a new product	Yes	363	80.7
	No	87	19.3

Know environmental problem of poor solid waste handling	Yes	373	82.9
	No	77	17.1

Know human health problems related to poor solid waste handling practices	Yes	405	90
	No	45	10

Type of health problems respondents knew related to poor solid waste handling	Malaria	341	75.8
	Cholera	244	54.2
	Typhoid	402	89.3
	Others	83	18.4

Knowing drinking water sources could be contaminated by solid wastes	Yes	369	82.0
	No	81	18.0

Know personal protective equipment used to handle solid waste?	Yes	412	91.6
	No	38	8.4

Overall knowledge	Good	226	50.2
	Poor	224	49.8

*Note.* ^*∗*^Others include skin and respiratory health problems.

The article "On-Site Solid Waste Handling Practice and Associated Factors among Condominium Residents in Gondar City, Northwest Ethiopia, 2021: A Community-Based Cross-Sectional Study" was published in 2023. Journal: J Environ Public Health.

**Table 3:** Attitude of condominium residents towards on-site solid waste handling practices in Gondar city, northwest Ethiopia, 2021.

Question items	Categories	Frequencies	Percentages (%)
Each person should manage his/her waste	Agree	62	13.8
	Disagree	388	86.2

I believe that poor solid waste disposal can cause air pollution	Agree	409	90.9
	Disagree	41	9.1

I believe that poor solid handling can cause human health problem	Agree	403	89.6
	Disagree	47	10.4

I am responsible to separate the waste I generated	Agree	423	94.0
	Disagree	27	6.0

I believe that waste recycling is very important	Agree	357	79.3
	Disagree	93	20.7

I always try to reduce the amount of solid waste I am producing	Agree	411	91.3
	Disagree	39	8.7

I believe that proper handling of solid waste can save money	Agree	380	84.4
	Disagree	70	15.6

Overall attitude	Favorable	191	42.4
	Unfavorable	259	57.6

**Table 4:** Infrastructural and institution-related factors of condominium residents towards on-site solid waste handling practices in Gondar city, northwest Ethiopia, 2021.

Variables	Frequencies	Percentages (%)
Access to streets to solid waste collectors between buildings		
Yes	216	48.0
No	234	52.0
Training regarding on-site solid waste handling practices		
Yes	67	14.9
No	383	85.1
Access to solid waste storage containers		
Yes	447	99.3
No	3	0.7
Legal control over a community to keep good solid waste handling		
Yes	312	69.3
No	138	30.7
Access to dry garbage for solid waste disposal		
Yes	423	94.0
No	27	6.0
Government has a budget for managing solid wastes from condominium		
Yes	399	88.7
No	51	11.3

**Table 5:** On-site solid waste handling practices among condominium residents in Gondar city, northwest Ethiopia, 2021 (*n* = 450).

Question items	Categories	Frequencies	Percentages (%)
Separate solid waste at home	Yes	377	83.8
	No	73	16.2

Reuse solid waste at home	Yes	34	7.6
	No	416	92.4

Recycle solid waste at home	Yes	42	9.3
	No	408	90.7

Store solid waste in a container	Yes	435	96.7
	No	15	3.3

Type of solid waste storage container at home	Plastics	114	25.3
	Sack	271	60.2
	Basket	65	14.4

Frequency of solid waste collection per week	Once	434	96.4
	Twice	16	3.6

Dump solid waste on the road	Yes	58	12.9
	No	392	87.1

Dump solid waste on the ditch	Yes	26	5.8
	No	424	94.2

Dump solid waste in the yard	Yes	28	6.2
	No	422	93.8

Burn SW in the compound	Yes	82	18.2
	No	368	81.8

Keep SW far from food	Yes	395	87.8
	No	55	12.2

Keep SW far from water	Yes	379	84.2
	No	71	15.8

Keep SW far away from children's playgrounds	Yes	421	93.6
	No	29	6.4

Overall on-site handling practice	Good	91	20.2
	Poor	359	79.8

The article "On-Site Solid Waste Handling Practice and Associated Factors among Condominium Residents in Gondar City, Northwest Ethiopia, 2021: A Community-Based Cross-Sectional Study" was published in 2023. Journal: J Environ Public Health.

**Table 6:** Bivariate and multivariable analysis of factors associated with on-site solid waste handling practices among condominium residents in Gondar city, northwest Ethiopia, 2021

Variables	On-site solid waste handling practices		COR (95%CI)	AOR (95%CI)
	Poor	Good		
Age of household heads				
>41	76 (81.7%)	17 (18.3%)	0.89 (0.43, 1.80)	0.99 (0.42, 2.36)
35–40	98 (76.6%)	30 (23.4%)	0.65 (0.34, 1.22)	0.64 (0.32, 1.36)
29–34	84 (77.8%)	24 (22.2%)	0.69 (0.36, 1.34)	0.79 (0.38, 1.65)
<29	101 (83.5%)	20 (16.5%)	1.00	1.00
Sex of household heads				
Male	177 (83.5%)	35 (16.5%)	1.56 (0.97, 2.49)	1.90 (1.11, 3.28)^*∗*^
Female	182 (76.5%)	56 (23.5%)	1.00	1.00
Educational status the household heads				
No formal education	43 (82.7%)	9 (17.3%)	1.24 (0.58, 2.65)	1.17 (0.49, 2.80)
Formal education	316 (79.4%)	82 (20.6%)	1.00	1.00
Monthly income				
>9001	46 (67.6%)	22 (32.4%)	0.50 (0.26, 0.96)	0.70 (0.30, 1.58)
7001–9000	75 (78.9%)	20 (21.1%)	0.89 (0.47, 1.70)	0.88 (0.38, 1.98)
5000–7000	117 (85.4%)	20 (14.6%)	1.40 (0.75, 2.62)	1.64 (0.88, 3.29)
<5000	121(80.7%)	29 (19.3%)	1.00	1.00
Family size				
5–8 members	**116 (85.3%)**	**20 (14.7%)**	**1.70 (0.98, 2.92)**	**1.87 (1.03, 3.40)** ^*∗*^
1–4 members	243 (77.4%)	71 (22.6%)	1.00	1.00
Occupational status of household head				
Government	158 (75.2%)	52 (24.8%)	0.72(0.43, 1.22)	0.66 (0.36, 1.20)
Private work	87 (87.9%)	12 (12.1%)	1.72 (0.82, 3.58)	1.74 (0.77, 3.94)
Housewife	114 (80.9%)	27 (19.1%)	1.00	1.00
Knowledge of on-site solid waste handling practices				
Poor	183 (81.7%)	41 (18.3%)	1.27(0.80, 2.01)	1.62 (0.92, 2.83)
Good	176 (77.9%)	50 (22.1%)	1.00	1.00
Attitude towards on-site solid waste handling practices				
Unfavorable	**218 (84.2%)**	**41 (15.8%)**	**1.89 (1.19, 2.99)**	**1.79 (1.07, 3.00)** ^*∗*^
Favorable	141 (73.8%)	50 (26.2%)	1.00	1.00
Training on on-site solid waste handling practices				
No	**318 (83.0%)**	**65 (17.0%)**	**3.10 (1.77, 5.43)**	**3.40 (1.77, 6.55)** ^*∗∗∗*^
Yes	41 (61.2%)	26 (38.8%)	1.00	1.00
Legal enforcement to keep proper on-site solid waste handling practices				
No	**121 (87.7%)**	**17 (12.3%)**	**2.21 (1.25, 3.92)**	**2.85 (1.39, 5.84)** ^*∗∗*^
Yes	238 (76.3%)	74 (23.7%)	1.00	1.00

*Note.* ^*∗*^ *p* value <0.05, ^*∗∗*^*p* value <0.01, ^*∗∗∗*^*p* value <0.001, model fitness test: 0.21, i.e., *p* < 0.05, and variance influence factors (VIF) test: <2, i.e., VIF <10.

## Data Availability

All data are available from the corresponding author.
